# A Novel Image Encryption Technique Based on Mobius Transformation

**DOI:** 10.1155/2021/1912859

**Published:** 2021-12-17

**Authors:** Muhammad Asif, Sibgha Mairaj, Zafar Saeed, M. Usman Ashraf, Kamal Jambi, Rana Muhammad Zulqarnain

**Affiliations:** ^1^Department of Mathematics, University of Management and Technology, Sialkot Campus, Sialkot, Pakistan; ^2^Department of Mathematics, University of Sialkot, Sialkot, Pakistan; ^3^Faculty of Information Technology, University of Central Punjab, Lahore, Pakistan; ^4^Department of Computer Science, University of Management and Technology, Sialkot Campus, Sialkot, Pakistan; ^5^Department of Computer Science, King Abdulaziz University, Jeddah, Saudi Arabia

## Abstract

The nonlinear transformation concedes as S-box which is responsible for the certainty of contemporary block ciphers. Many kinds of S-boxes are planned by various authors in the literature. Construction of S-box with a powerful cryptographic analysis is the vital step in scheming block cipher. Through this paper, we give more powerful and worthy S-boxes and compare their characteristics with some previous S-boxes employed in cryptography. The algorithm program planned in this paper applies the action of projective general linear group *PGL*(2, *GF*(2^8^)) on Galois field *GF*(2^8^). The proposed S-boxes are constructed by using Mobius transformation and elements of Galois field. By using this approach, we will encrypt an image which is the preeminent application of S-boxes. These S-boxes offer a strong algebraic quality and powerful confusion capability. We have tested the strength of the proposed S-boxes by using different tests, BIC, SAC, DP, LP, and nonlinearity. Furthermore, we have applied these S-boxes in image encryption scheme. To check the strength of image encryption scheme, we have calculated contrast, entropy, correlation, energy, and homogeneity. The results assured that the proposed scheme is better. The advantage of this scheme is that we can secure our confidential image data during transmission.

## 1. Introduction

The notion of S-box was first introduced by applied scientist Claude Shannon in 1949, and afterward this notion has attracted the attention of many researchers. With the quick evolution of the network communication and massive data application, the security of the data has become more popular topic. The scholars have proposed a spread of the information encryption, privacy protection. In symmetric cryptography, the block encryption algorithm is used customarily, for example, in encryption (DES), AES, and other systems. In block cipher system, there is a predominant nonlinear component called substitution box. S-box plays a crucial role in the security of symmetric cryptosystem. AES is taken into account to be an efficient cryptosystem to a large extent. One of the important components of the AES is its prime S-box which is predicted on the inversion and transformation because of recognition of AES in the communication system; substitution box captivates traditional attention. However, the substitution box which is employed in AES is predetermined. The S-box is a nonlinear component of block cipher which creates confusion. The maintenance of information security has become an excellent challenge for the cryptography. Substitution boxes have been employed in many cryptosystems including encryption standard (DES), international data encryption algorithm (IDEA), and advanced encryption standard (AES). The security strength of substitution box determines the safety of the entire cryptosystem. It is therefore established that the substitution box is the important nonlinear component of the cryptographic system. Cryptography has unprecedented ways of the utilization of encryption capabilities to produce security of the data.

Many image encryption algorithms with S-box have been presented [1–8]. Liu et al. [6] explained the image encryption scheme using one-time S-boxes. Hussain and Gondal [5] gave an extended image encryption using chaotic coupled map and S-box transformation, the confusion-diffusion structure was assumed, the places of the pixels of the plain image were mixed up by a chaotic tent map, and after that delayed coupled map lattices and S-box transformation were used to puzzle the association between the original image and the cipher image. Zhang et al. [9] introduced an efficient chaotic image encryption based on alternate circular S-boxes, and a set of S-boxes were constructed by Chen chaotic system. Liu et al. [10, 11] developed the adaptive controller design and fuzzy synchronization for uncertain fractional order nonlinear system and fractional order chaotic systems. The scrutiny of AES is explained considering the high throughput, area efficiency, and elevated performance [12]. Khan et al. [13] introduced an efficient image encryption scheme based on double affine substitution box and chaotic system. Asif and Shah [14] explained the image encryption scheme using BCH codes. Alanazi et al. [15] explained cryptanalysis of novel image encryption scheme based on multiple chaotic substitution boxes. An approach to increasing multimedia security employing 3D mixed chaotic map and hybrid permutation substitution is explained by Naseer et al. [16, 17]. Khalid et al. [18] defined elliptic curve based image encryption scheme by using S-boxes. Cryptanalysis on S-box based on encryption method is clarified by Munir et al. [19]. Nonlinear component based on elliptic curve and power associative loop structure is defined by Haider et al. [20] and Hussain et al. [21], respectively.

The above presented studies are not enough to secure data in communication channel. To overcome this drawback, we proposed a novel approach using Mobius transformation. Existing studies deal only with one S-box for AES algorithm, but our proposed scheme is utilized to encrypt image using ten S-boxes. The rest of the paper is organized as follows: The elements of S-box are constructed by using elements of Galois field in Section 2, and the elements of Galois field are utilized in linear fractional transformation for S-boxes. In Section 3, analysis of S-boxes is carried out, and comparison with other S-boxes is also made. In Section 4, image encryption scheme is proposed by utilizing S-boxes, different tests are applied on encrypted image, and comparison of image encryption scheme with existing techniques is provided. The conclusion of the paper is presented in Section 5.

## 2. Construction of S-Box Using Galois Field

### 2.1. Galois Field

Any finite field is called Galois field. Nowadays, Galois field is used in many cryptographic algorithms for data security. A Galois filed extension is defined as

(1) $$\begin{array}{c} GF\left(p^{m}\right)=\frac{Z_{p}\left[x\right]}{\langle f\left(x\right)\rangle }, \end{array}$$

where *f*(*x*) is primitive irreducible polynomial of degree *m*.

### 2.2. Scheme for Construction of S-Box

A 16 × 16 S-box is constructed using the elements of Galois field. The total elements of the proposed S-box are 256, which are constructed by the action of *PGL*(2, *GF*(2^8^)) on *GF*(2^8^) [22]. Now, we have the Mobius transformation:

(2) $$\begin{array}{c} T:\;PGL\left(2,\;GF\left(2^{8}\right)\right)\times GF\left(2^{8}\right)⟶GF\left(2^{8}\right),\\ T\left(t\right)=\frac{at+b}{ct+d}, \end{array}$$

where *a*, *b*, *c*, *d*, and *t* ∈ *GF*(2^8^).

Here, *T*(*t*) are the values of *GF*(2^8^) to construct the new S-box. This algorithm will stop working when *a*.*d* − *b*.*c* ≠ 0 does not exist. Moreover, after the change of the values in dividend and divisor, there is also a scenario where results of divisor are equal to zero. We additionally check this worth of unassisted degree rule that makes divisor zero; to overcome this type of error zero divisor, we assign the associated remaining value to conclude the values of substitution box. To find the elements, we substitute the value of *t* from 0 to 255 and convert *t*,  *a*,  *b*,  *c*,  *d* to binary form. Before control on the binary type, simply ones tend to delineate the values in form of polynomials. The terms from dividend and divisor of the unit being modified with the corresponding binary values “*m*” are interpreted as a particular primitive polynomial

(3) $$\begin{array}{c} P\left(x\right)=x^{8}+x^{4}+x^{3}+x^{2}+1. \end{array}$$

Here, *P*(*x*) is utilized for the construction of the elements of the *GF*(2^8^) [23]. The mathematical methodology for *GF*(2^8^) will be used in our further process. We can define *GF*(2^8^)=*ℤ*_2_[*x*]/〈*P*(*x*)〉, where *ℤ*_2_={0,1} and the polynomial *P*(*x*)=*x*^8^+*x*^4^+*x*^3^+*x*^2^+1 is the primitive irreducible polynomial.

Now, we construct the values of the transformed S-box by using Mobius transformation and elements of Galois field from Table 1. Here, we consider *a*=220, *b*=30, *c*=90,  and *d*=200,  where *t*=0 to 255.

(4) $$\begin{array}{c} T\left(t\right)=\frac{220\left(t\right)+30}{90\left(t\right)+200}. \end{array}$$

Here, *t*=0 to 255. We consider *t*=0; then,

(5) $$\begin{array}{c} T\left(0\right)=\frac{220\left(0\right)+30}{90\left(0\right)+200}. \end{array}$$

Converting each value into binary form, we will get the polynomial of the corresponding values. We can see the corresponding value of this polynomial in Table 1 in form of “*x*.”

(6) $$\begin{array}{c} T\left(0\right)=x^{7}+x^{5}+x^{3}+1=10101001=169. \end{array}$$

Therefore, the first value of the transformed S-box is 169; by following the same procedure, we will compute the remaining elements of the S-box.

## 3. Analysis of Transformed S-Boxes and Their Comparison Support

Nonlinearity constitutes the quantity of bits which are necessarily altered to succeed in affine at the lowest distance. Therefore, for an outsize “*m*,” that calculation is going to be difficult. Now, we will mention the series of the function on *Fⁿ* with *α*, so the nonlinearity is defined as

(7) $$\begin{array}{c} Nf=2^{n-1}\frac{1}{2_{\left\{i=0,1,2,3,\ldots ,2^{n-1}\right\}}}\max\left\{\left|\langle \alpha ,l_{\left\{i\right\}}\rangle \right|\right\}, \end{array}$$

(8) $$\begin{array}{c} B_{n}=\left(\begin{array}{cc} B_{n-1}\\ B_{n-1} & B_{n-1} \end{array}\right), \end{array}$$

The nonlinearity of these S-boxes should satisfy the following relation [24]:

(9) $$\begin{array}{c} N_{f}=\frac{2^{n}-2^{n/2}}{2}=120,\;\text{when }n=8, \end{array}$$

120 is considered as an absolute nonlinearity value.

From Tables 2–11, we observe that from Table 12 the maximum nonlinearity of transformed S-box is equal to 107.3, which is better when compared to other S-boxes.

### 3.1. Strict Avalanche Criterion (SAC)

A median consequence of the resulting bits should be modified to 0.5. Once one input bit is executed, then the given alteration shows associated avalanche result. The given operate clutch an effective avalanche result if the method is replicate for all input bits also almost 50%  avalanche variable attain value 1. S-box fulfills the SAC if only 1 input bit is modified so that in the result 0.5 quantities of output bits are changed. For the function expression, *f*(*x*) ⊕ *f*(*x* ⊕ *α*) is safe for the sequence *α* such that the weight of the *α*=1, so the function *f* :  *F*_2_^*n*^⟶*F*_2_ fulfills SAC [29].

By considering the maximum values and minimum values, we observe that the average value of SAC from Table 13 is comparatively better and ∼0.5.

### 3.2. Bit Independence Criterion (BIC)

This is another style of criterion for the S-box to calculate the worth outlined because the output *Y* and *Z* should be altered separately. A bit independence criterion is an appropriate property for each crypt analytical scheme, which was introduced by Webster and Tavares. It has been argued that the Boolean functions *f*_*y*_, *f*_*z*_(*y* ≠ *z*) are two different output bits of the S-box. If S-box encounters bit independence criterion, *f*_*y*_ ⊕ *f*_*z*_(*y* ≠ *z*, 1 ≤ *y*, *z* ≤ *n*) should be exceptionally nonlinear and are available as near as possible in order to satisfy strict avalanche criterion. We are able to conjointly attest the bit independence by evaluating nonlinearity and strict avalanche criterion of *f*_*y*_ ⊕ *f*_*z*_ [30].

In Table 14 for comparison of BIC, we take minimum value; our minimum value is 101.3, which is better compared to *S*_8_ Liu J, Hussain et al., and residue prime S-boxes.

### 3.3. Linear Approximation Probability (LP)

It is determined as the highest worth of inequality of a happening. The uniformity of input bits should be the image of the uniformity of the output bits. At the level of input *i*^th^, input bit is evaluated severally and also its consequences part discovered within the output bits formula where 2^*m*^ shows the quantity of pats belong to the constructed S-box and also the assortment of every feasible input bits to S-box, part is denoted by *X*, where Φ(*x*) and Φ(*y*) show input/output [15].

Table 15 shows that our transformed S-box against linear attacks is better when compared to residue prime S-box and identical to Hussain S-box.

### 3.4. Differential Approximation Probability (DP)

The S-box is considered because it is a nonlinear component of block cipher. In the perfect situation, S-box shows the different consistency. Δ*x* is considered as the input differential whereas Δ*y* indicates the output differential. During the technique of immigrant, it has been noticed, what quantity chance that differential of the input bits is is separately mapped on differential at output bits. Associate degree input differential associated degree should separately map to output Δ*y*. To calculate the differential uniformity, the DP of specified S-box can be explicit as follows:

(10) $$\begin{array}{c} DP\left(\Delta x,\;\Delta y\right)=\frac{\text{number of}\left\{x\in X╱S\left(x\right)⊕S\left(x⊕\Delta x\right)=\Delta y\right\}}{2^{m}}. \end{array}$$

Here, *x* represents a set of the possible feasible input values and their number of components are denoted by 2^*m*^.

Table 16 shows that S-box maintains its maximum differential probability at 0.06 which is acceptable value for resistance against differential attacks.

## 4. Application of the Proposed S-Boxes

The most advanced encryption standard algorithm is used for image encryption data. We can encrypt any image by using AES in MATLAB. We will not get any information of the original image when the image is encrypted. From this, we can see that AES encryption algorithm can get the results of image encryption. The AES encryption system is symmetric; it has three types of key length of encryption: 128, 196, and 256 bits, with a packet size of 128 bits for all; and the algorithm has fantastic flexibility. Therefore, it is being used in software and also in hardware. In this 3-key length of AES algorithm, 128 bits' key length is commonly used. Under this key length, 10-time iterative computation is done in the internal algorithm. Additionally, in the final round, every round contains five portions: Sub Bytes, S-box, Shift Rows, Mix Columns, and Add Round Key. Here, we perform the digital image encryption and will get the date which uses encryption algorithm of AES. Then, digital image encrypted by using AES algorithm is realized in the MATLAB simulation.

From Figure 1, we can see that the host image is unpredictable when performing 1st round of AES, and this disorder in the picture increases as we perform other rounds. The feature of the image can also be described through gray histogram of image, which shows the number of occurrences of different pixel values. If the image contains a low contrast, then histogram will be narrow and will be focused in the middle of gray scale. From the result, it has been clear that AES algorithm has excellent effect for the encrypted image.

### 4.1. Majority Logic Criterion for S-Boxes

The majority logic criterion is applicable within the evaluation procedure of S-boxes, employed in AES (advanced encryption standard). The strength of the proposed S-boxes is checked by statistical analyses. The essential component of statistical analysis used for the sake of majority logic criterion is derived from the results of the following:

- Contrast
- Correlation
- Energy
- Homogeneity
- Entropy

In the process of substitution, firstly data is altered into the form of encrypted data. On the other side, within the permutation process, the order of data material or contents is changed, which results in a different arrangement of the bits. The process of the substitution depends on the quantity of bits' n which makes the number of keys equal to 2ⁿ. The amalgamation of the permutation and the substitution of the data bit at the level of input make the encryption of the data stronger.

#### 4.1.1. Contrast

The bulk of the contrast within the picture allows the viewer to brightly identify objects in a picture. Because the picture is encrypted, the amount of disorderness increases; as a result, it elevates the level of contrast to a really high value. Contrast is actually associated with the quantity of confusion which is created by the S-box within the original image. The mathematical depiction of contrast analysis is

(11) $$\begin{array}{c} \text{contrast}=\sum {\left|i-j\right|}^{2}p\left(i,j\right). \end{array}$$

Here *i*, *j* denotes the pixels of the image.  Figure 2 shows the illustration of contrast.

#### 4.1.2. Correlation

Correlation elaborates the relation between the pixels in the image data. Correlation analysis is split into three different parts. It is performed on the following:

- Vertical and horizontal
- Diagonal formats
- General correlation

Additionally, for analysis on a partial region, the complete image is additionally included within the processing. This analysis calculates the correlation of the pixel to its neighbor by taking into consideration the pixels of complete image data.

If *M, N* identifies two matrix and *M_mn_, N_mn_* identifies the mean of the matrix elements, the for correlation is

(12) $$\begin{array}{c} \text{correlation}=\sqrt{\frac{\sum_{m}\sum_{n}\left(M_{mn}-\bar{M}\right)\left(N_{mn}-\bar{N}\right)}{\sum_{m}\sum_{n}{\left(M_{mn}-\bar{M}\right)}^{2}\sum_{m}\sum_{n}{\left(N_{mn}-\bar{N}\right)}^{2}}}. \end{array}$$

The correlation of the same image is one bit; if the correlations are equal, this does not mean that photographs are the same. Two different pictures may have the same correlation, but distribution of the pixel colors might be completely distinct as shown in Figure 3.

#### 4.1.3. Energy

The analysis of energy is employed to measure the encrypted image. The gray-level cooccurrence matrix is employed to conduct energy. The performance of previous substitution box is healthier than the previous S-box utilized in analysis. The mathematical representation of the energy is

(13) $$\begin{array}{c} \text{energy}=\sum P{\left(i,j\right)}^{2}. \end{array}$$

#### 4.1.4. Homogeneity

The data of image contains a natural distribution that is related to the contents of the corresponding image. We execute the homogeneity which calculates the closeness of the distributed components. This is often called gray-tone spatial dependency matrix. The GLCM represents the combination of the pixel brightness values or the gray-levels that are formed in a table. The frequency of gray levels is often illuminated from the table GLCM.

The homogeneity is often determined as

(14) $$\begin{array}{c} \sum_{ij}\frac{p\left(i,j\right)}{1+\left|i-j\right|}. \end{array}$$

Here, gray level cooccurrence matrices in the GLCM are mentioned by *P*(*i*, *j*).

#### 4.1.5. Entropy

Entropy is often defined because of the randomness in the picture. The entropy of encrypted image is denoted as

(15) $$\begin{array}{c} \text{entropy}=-\sum_{i=1}^{n}\left(p\left(x_{i\;}\right)\log_{b}p\left(x_{i}\right)\right), \end{array}$$

where *p*(*x*_*i* _) have the histogram count.  Figure 4 shows the comparison of higher and lower entropy. A superbly random image entropy has the value 8. Because the image gets foreseeable, entropy decreases. Therefore, in order to get good encrypted image, entropy must be closest to 8.

Here, Table 17 shows the majority logic criterion of S-boxes which satisfy all the criteria up to standard that can be used for the sake of communication.

The entropy measures the strength of image encryption scheme. If entropy is nearly equal to 8, this means that our image encryption scheme is good. If contrast is high, the strength of the encrypted image is more beneficial. Correlation close to zero as much as possible shows better encrypted image quality. If energy and homogeneity decrease and approximately equal zero, then the proposed image encryption scheme is better.

Table 17 shows that entropy of encrypted image is close to 8, contrast is very high, correlation and energy are close to zero, and homogeneity also decreases. From these tests and comparisons, we can say that the proposed image encryption scheme using 10 different S-boxes in different round is very good.

## 5. Conclusion

S-box is the consequential component in the algorithm of encryption melded into SPN that plays a crucial part. In this work, we utilize a technique for the construction of worthy S-box which is established because of the action of *PGL*(2, *GF*(2^8^)) on a Galois field *GF*(2^8^). This new constructed S-box relates to a special sort of Mobius transformation. It has been observed from the appraisal that representation scheme of new S-box is undemanding and straightforward for the software and hardware application. Furthermore, to analyze the capability of S-box, we have applied different tests, nonlinearity, BIC, SAC, LP, and DP. Then, we have used these S-boxes in image encryption and checked the strength of image encryption by applying different tests, contrast, correlation, entropy, energy, and homogeneity. We have compared the results with others; hence, we conclude that the proposed scheme produces efficient results compared to other ones. The comparison of LP, DP, strict avalanche criterion, and bit independence criterion with existing techniques assured that the proposed scheme for image encryption is better. In future, proposed S-boxes will be used for audio, video, and text encryption scheme. Proposed image encryption scheme is used for data security of different military intelligence agencies.

## Figures and Tables

**Figure 1:** Image encryption with histogram analysis.

**Figure 2:** Illustration of contrast.

**Figure 3:** Correlation of encrypted image.

**Figure 4:** Higher vs. lower entropy.

**Table 1:** Elements of Galois field *GF*(2^8^).

Exp.	Decimal	Polynomial
*x* ^0^	01	*x* ^0^
*x* ^1^	02	*x* ^1^
*x* ^2^	04	*x* ^2^
*x* ^3^	08	*x* ^3^
*x* ^4^	16	*x* ^4^
*x* ^5^	32	*x* ^5^
*x* ^6^	64	*x* ^6^
*x* ^7^	128	*x* ^7^
*x* ^8^	29	*x* ^4^+*x*^3^+*x*^2^+1
*x* ^9^	58	*x* ^5^+*x*^4^+*x*^3^+*x*
*x* ^10^	116	*x* ^6^+*x*^5^+*x*^4^+*x*^2^
*x* ^11^	232	*x* ^7^+*x*^6^+*x*^5^+*x*^3^
*x* ^12^	205	*x* ^7^+*x*^6^+*x*^3^+*x*^2^+1
*x* ^13^	135	*x* ^7^+*x*^2^+*x*+1
*x* ^14^	19	*x* ^4^+*x*+1
*x* ^15^	38	*x* ^5^+*x*^2^+*x*
*x* ^16^	76	*x* ^6^+*x*^3^+*x*^2^
*x* ^17^	152	*x* ^7^+*x*^4^+*x*^3^
*x* ^18^	45	*x* ^5^+*x*^3^ + *x*^2^+1
*x* ^19^	90	*x* ^6^+*x*^4^+*x*^3^+*x*
*x* ^20^	180	*x* ^7^+*x*^5^+*x*^4^+*x*^2^
*x* ^21^	117	*x* ^6^+*x*^5^+*x*^4^+*x*^2^+1
*x* ^22^	234	*x* ^7^+*x*^6^+*x*^5^+*x*^3^+*x*
*x* ^23^	201	*x* ^7^+*x*^6^+*x*^3^+1
*x* ^24^	143	*x* ^7^+*x*^3^+*x*^2^+*x*+1
*x* ^25^	3	*x*+1
*x* ^26^	6	*x* ^2^+*x*
*x* ^27^	12	*x* ^3^+*x*^2^
*x* ^28^	24	*x* ^4^+*x*^3^
*x* ^29^	48	*x* ^5^+*x*^4^
*x* ^30^	96	*x* ^6^+*x*^5^
*x* ^31^	192	*x* ^7^+*x*^6^
*x* ^32^	157	*x* ^8^+*x*^7^
*x* ^33^	39	*x* ^5^+*x*^2^+*x*+1
*x* ^34^	78	*x* ^6^+*x*^3^+*x*^2^+*x*
*x* ^35^	156	*x* ^7^+*x*^4^+*x*^3^+*x*^2^
*x* ^36^	37	*x* ^5^+*x*^2^+1
*x* ^37^	74	*x* ^6^+*x*^3^+*x*
*x* ^38^	148	*x* ^7^+*x*^4^+*x*^2^
*x* ^39^	53	*x* ^5^+*x*^4^+*x*^2^+1
*x* ^40^	106	*x* ^6^+*x*^5^+*x*^3^+*x*
*x* ^41^	212	*x* ^7^+*x*^6^+*x*^4^+*x*^2^
*x* ^42^	181	*x* ^7^+*x*^5^+*x*^4^+*x*^2^+1
*x* ^43^	119	*x* ^6^+*x*^5^+*x*^4^+*x*^2^+*x*+1
*x* ^44^	238	*x* ^7^+*x*^6^+*x*^5^+*x*^3^+*x*^2^+*x*
*x* ^45^	193	*x* ^7^+*x*^6^+1
*x* ^46^	159	*x* ^7^+*x*^4^+*x*^3^+*x*^2^+*x*+1
*x* ^47^	35	*x* ^5^+*x*+1
*x* ^48^	70	*x* ^6^+*x*^2^+*x*
*x* ^49^	140	*x* ^7^+*x*^3^+*x*^2^
*x* ^50^	5	*x* ^2^+1
*x* ^51^	10	*x* ^3^+*x*
*x* ^52^	20	*x* ^4^+*x*^2^
*x* ^53^	40	*x* ^5^+*x*^3^
*x* ^54^	80	*x* ^6^+*x*^4^
*x* ^55^	160	*x* ^7^+*x*^5^
*x* ^56^	93	*x* ^6^+*x*^4^+*x*^3^+*x*^2^+1
*x* ^57^	186	*x* ^7^+*x*^5^+*x*^4^+*x*^3^+*x*
*x* ^58^	105	*x* ^6^+*x*^5^+*x*^3^+1
*x* ^59^	210	*x* ^7^+*x*^6^+*x*^4^+*x*
*x* ^60^	185	*x* ^7^+*x*^5^+*x*^4^+*x*^3^+1
*x* ^61^	111	*x* ^6^+*x*^5^+*x*^3^+*x*^2^+*x*+1
*x* ^62^	223	*x* ^7^+*x*^6^+*x*^4^+*x*^3^+*x*^2^+*x*
*x* ^63^	161	*x* ^7^+*x*^5^+1
*x* ^64^	95	*x* ^6^+*x*^4^+*x*^3^+*x*^2^+*x*+1
*x* ^65^	190	*x* ^7^+*x*^5^+*x*^4^+*x*^3^+*x*^2^+*x*
*x* ^66^	97	*x* ^6^+*x*^5^+1
*x* ^67^	194	*x* ^7^+*x*^6^+*x*
*x* ^68^	153	*x* ^7^+*x*^4^+*x*^3^+1
*x* ^69^	47	*x* ^5^+*x*^4^+*x*^2^+*x*+1
*x* ^70^	94	*x* ^6^+*x*^4^+*x*^3^+*x*^2^+*x*
*x* ^71^	188	*x* ^7^+*x*^5^+*x*^4^+*x*^3^+*x*^2^
*x* ^72^	101	*x* ^6^+*x*^5^+*x*^2^+1
*x* ^73^	202	*x* ^7^+*x*^6^+*x*^3^+*x*
*x* ^74^	137	*x* ^7^+*x*^3^+1
*x* ^75^	15	*x* ^3^+*x*^2^+*x*+1
*x* ^76^	30	*x* ^4^+*x*^3^+*x*^2^+*x*
*x* ^77^	60	*x* ^5^+*x*^4^+*x*^3^+*x*^2^
*x* ^78^	120	*x* ^6^+*x*^5^+*x*^4^+*x*^3^
*x* ^79^	240	*x* ^7^+*x*^6^+*x*^5^+*x*^4^
*x* ^80^	253	*x* ^7^+*x*^6^+*x*^5^+*x*^4^+*x*^3^+*x*^2^+1
*x* ^81^	231	*x* ^7^+*x*^6^+*x*^5^+*x*^2^+*x*+1
*x* ^82^	211	*x* ^7^+*x*^6^+*x*^2^+*x*+1
*x* ^83^	187	*x* ^7^+*x*^5^+*x*^4^+*x*^3^+*x*+1
*x* ^84^	107	*x* ^6^+*x*^5^+*x*^3^+*x*+1
*x* ^85^	214	*x* ^7^+*x*^6^+*x*^4^+*x*^2^+*x*
*x* ^86^	177	*x* ^7^+*x*^5^+*x*^4^+1
*x* ^87^	127	*x* ^6^+*x*^5^+*x*^4^+*x*^3^+*x*^2^+*x*+1
*x* ^88^	254	*x* ^7^+*x*^6^+*x*^5^+*x*^4^+*x*^3^+*x*^2^+*x*
*x* ^89^	225	*x* ^7^+*x*^6^+*x*^5^+1
*x* ^90^	223	*x* ^7^+*x*^6^+*x*^4^+*x*^3^+*x*^2^+*x*+1
*x* ^91^	163	*x* ^7^+*x*^5^+*x*+1
*x* ^92^	91	*x* ^6^+*x*^4^+*x*^3^+*x*^3^+*x*+1
*x* ^93^	182	*x* ^7^+*x*^5^+*x*^4^+*x*^2^+*x*
*x* ^94^	113	*x* ^6^+*x*^5^+*x*^4^+1
*x* ^95^	226	*x* ^7^+*x*^6^+*x*^3^+*x*
*x* ^96^	217	*x* ^7^+*x*^6^+*x*^4^+*x*^3^+1
*x* ^97^	175	*x* ^7^+*x*^5^+*x*^3^+*x*^2^+*x*+1
*x* ^98^	67	*x* ^6^+*x*+1
*x* ^99^	134	*x* ^7^+*x*^2^+*x*
*x* ^100^	17	*x* ^4^+1
*x* ^101^	34	*x* ^5^+*x*
*x* ^102^	68	*x* ^6^+*x*^2^
*x* ^103^	136	*x* ^7^+*x*^3^
*x* ^104^	13	*x* ^3^+*x*^2^+1
*x* ^105^	26	*x* ^4^+*x*^3^+*x*
*x* ^106^	152	*x* ^5^+*x*^4^+*x*^2^
*x* ^107^	104	*x* ^6^+*x*^5^+*x*^3^
*x* ^108^	208	*x* ^7^+*x*^6^+*x*^4^
*x* ^109^	189	*x* ^8^+*x*^7^+*x*^5^
*x* ^110^	103	*x* ^6^+*x*^5^+*x*^2^+*x*+1
*x* ^111^	206	*x* ^7^+*x*^6^+*x*^3^+*x*^2^+*x*
*x* ^112^	129	*x* ^7^+1
*x* ^113^	31	*x* ^4^+*x*^3^+*x*^2^+*x*+1
*x* ^114^	62	*x* ^5^+*x*^4^+*x*^3^+*x*^2^+*x*
*x* ^115^	124	*x* ^6^+*x*^5^+*x*^4^+*x*^3^+*x*^2^
*x* ^116^	248	*x* ^7^+*x*^6^+*x*^5^+*x*^4^+*x*^3^
*x* ^117^	237	*x* ^7^+*x*^6^+*x*^5^+*x*^3^+*x*^2^+1
*x* ^118^	199	*x* ^7^+*x*^6^+*x*^2^+*x*+1
*x* ^119^	147	*x* ^7^+*x*^4^+*x*+1
*x* ^120^	59	*x* ^5^+*x*^4^+*x*^3^+*x*+1
*x* ^121^	118	*x* ^6^+*x*^5^+*x*^4^+*x*^2^+*x*
*x* ^122^	236	*x* ^7^+*x*^6^+*x*^5^+*x*^3^+*x*^2^
*x* ^123^	197	*x* ^7^+*x*^6^+*x*^2^+1
*x* ^124^	151	*x* ^7^+*x*^4^+*x*^2^+*x*+1
*x*^125^	51	*x* ^5^+*x*^4^+*x*+1
*x*^126^	102	*x* ^6^+*x*^5^+*x*^2^+*x*
*x* ^127^	204	*x* ^7^+*x*^6^+*x*^3^+*x*^2^
*x* ^128^	133	*x* ^7^+*x*^2^++1
*x* ^129^	23	*x* ^4^+*x*^2^+*x*+1
*x* ^130^	46	*x* ^5^+*x*^3^+*x*^2^+*x*
*x* ^131^	92	*x* ^6^+*x*^4^+*x*^3^+*x*^2^
*x* ^132^	184	*x* ^7^+*x*^5^+*x*^4^+*x*^3^
*x*^133^	109	*x* ^6^+*x*^5^+*x*^3^+*x*^2^+1
*x*^134^	218	*x* ^7^+*x*^6^+*x*^4^+*x*^3^+*x*
*x*^135^	169	*x* ^7^+*x*^5^+*x*^3^+1
*x*^136^	47	*x* ^6^+*x*^3^+*x*^2^+*x*+1
*x*^137^	94	*x* ^7^+*x*^4^+*x*^3^+*x*^2^+*x*
*x* ^138^	188	*x* ^5^+1
*x* ^139^	66	*x* ^6^+*x*
*x* ^140^	132	*x* ^7^+*x*^2^
*x* ^141^	21	*x* ^4^+*x*^2^+1
*x* ^142^	42	*x* ^5^+*x*^3^+*x*
*x* ^143^	84	*x* ^6^+*x*^4^+*x*^2^
*x* ^144^	168	*x* ^7^+*x*^5^+*x*^3^
*x* ^145^	77	*x* ^6^+*x*^3^+*x*^2^+1
*x* ^146^	154	*x* ^7^+*x*^4^+*x*^3^+*x*
*x* ^147^	41	*x* ^5^+*x*^3^+1
*x* ^148^	82	*x* ^6^+*x*^4^+*x*
*x* ^149^	164	*x* ^7^+*x*^5^+*x*^2^
*x* ^150^	85	*x* ^6^+*x*^4^+*x*^2^
*x* ^151^	170	*x* ^7^+*x*^5^+*x*^3^+*x*
*x* ^152^	73	*x* ^6^+*x*^3^+1
*x*^153^	146	*x* ^7^+*x*^4^+*x*
*x* ^154^	57	*x* ^5^+*x*^4^+*x*^3^+1
*x* ^155^	114	*x* ^6^+*x*^5^+*x*^4^+*x*
*x* ^156^	228	*x* ^7^+*x*^6^+*x*^5^+*x*^2^
*x* ^157^	213	*x* ^7^+*x*^6^+*x*^4^+*x*^2^+1
*x* ^158^	183	*x* ^7^+*x*^5^+*x*^4^+*x*^2^+*x*+1
*x* ^159^	115	*x* ^6^+*x*^5^+*x*^4^+*x*+1
*x* ^160^	230	*x* ^7^+*x*^6^+*x*^5^+*x*^2^+*x*
*x* ^161^	209	*x* ^7^+*x*^6^+*x*^4^+1
*x* ^162^	191	*x* ^7^+*x*^5^+4+*x*^3^+*x*^2^+*x*+1
*x* ^163^	99	*x* ^6^+*x*^5^+*x*+1
*x* ^164^	198	*x* ^7^+*x*^6^+*x*^2^+*x*
*x* ^165^	145	*x* ^7^+*x*^4^+1
*x* ^166^	63	*x* ^5^+*x*^4^+*x*^3^+*x*^2^+*x*+1
*x* ^167^	126	*x* ^6^+*x*^5^+*x*^4^+*x*^3^+*x*^2^+*x*
*x* ^168^	252	*x* ^7^+*x*^6^+*x*^5^+*x*^4^+*x*^3^+*x*^2^
*x* ^169^	229	*x* ^7^+*x*^6^+*x*^5^+*x*^2^
*x* ^170^	215	*x* ^7^+*x*^6^+*x*^4^+*x*^4^+*x*+1
*x* ^171^	179	*x* ^7^+*x*^5^+*x*^4^+*x*+1
*x* ^172^	123	*x* ^6^+*x*^5^+*x*^4^+*x*^3^+*x*+1
*x* ^173^	246	*x* ^7^+*x*^6^+*x*^5^+*x*^4^+*x*^2^+*x*
*x* ^174^	241	*x* ^7^+*x*^6^+*x*^5^+*x*^4^+1
*x* ^175^	255	*x* ^7^+*x*^6^+*x*^5^+*x*^4^+*x*^3^+*x*^2^+*x*+1
*x* ^176^	227	*x* ^7^+*x*^6^+*x*^5^+*x*+1
*x* ^177^	219	*x* ^7^+*x*^6^+*x*^4^+*x*^3^+*x*+1
*x* ^178^	171	*x* ^7^+*x*^5^+*x*^3^+*x*+1
*x* ^179^	75	*x* ^6^+*x*^3^+*x*+1
*x* ^180^	150	*x* ^7^+*x*^4^+*x*^2^+*x*
*x* ^181^	49	*x* ^5^+*x*^4^+1
*x* ^182^	98	*x* ^6^+*x*^5^+*x*
*x* ^183^	196	*x* ^7^+*x*^6^+*x*^2^
*x* ^184^	149	*x* ^7^+*x*^4^+*x*^2^+1
*x* ^185^	55	*x* ^5^+*x*^4^+*x*^2^+*x*+1
*x* ^186^	110	*x* ^6^+*x*^5^+*x*^3^+*x*^2^+*x*
*x*^187^	220	*x* ^7^+*x*^6^+*x*^4^+*x*^3^+*x*^2^
*x* ^188^	165	*x* ^7^+*x*^5^+*x*^2^+1
*x* ^189^	87	*x* ^6^+*x*^4^+*x*^2^+*x*+1
*x* ^190^	174	*x* ^7^+*x*^5^+*x*^3^+*x*^2^+*x*
*x* ^191^	65	*x* ^6^+1
*x* ^192^	130	*x* ^7^+*x*
*x* ^193^	25	*x* ^4^+*x*^3^+1
*x* ^194^	50	*x* ^5^+*x*^4^+*x*
*x* ^195^	100	*x* ^6^+*x*^5^+*x*^2^
*x* ^196^	200	*x* ^7^+*x*^6^+*x*^3^
*x* ^197^	141	*x* ^7^+*x*^3^+*x*^2^+1
*x* ^198^	7	*x* ^2^+*x*+1
*x* ^199^	14	*x* ^3^+*x*^2^+*x*
*x* ^200^	28	*x* ^4^+*x*^3^+*x*^2^
*x* ^201^	56	*x* ^5^+*x*^4^+*x*^3^
*x* ^202^	112	*x* ^6^+*x*^5^+*x*^4^
*x* ^203^	224	*x* ^7^+*x*^6^+*x*^5^
*x* ^204^	221	*x* ^7^+*x*^6^+*x*^4^+*x*^3^+*x*^2^+1
*x* ^205^	167	*x* ^7^+*x*^5^+*x*^2^+*x*+1
*x* ^206^	83	*x* ^6^+*x*^4^+*x*+1
*x* ^207^	166	*x* ^7^+*x*^5^+*x*^2^+*x*
*x* ^208^	81	*x* ^6^+*x*^4^+1
*x* ^209^	162	*x* ^7^+*x*^5^+*x*
*x* ^210^	89	*x* ^6^+*x*^4^+*x*^3^+1
*x* ^211^	178	*x* ^7^+*x*^5^+*x*^4^+*x*
*x* ^212^	121	*x* ^6^+*x*^5^+*x*^4^+*x*^3^+1
*x* ^213^	242	*x* ^7^+*x*^6^+*x*^5^+*x*^4^+*x*
*x* ^214^	249	*x* ^7^+*x*^6^+*x*^5^+*x*^4^+*x*^3^+1
*x* ^215^	239	*x* ^7^+*x*^6^+*x*^5^+*x*^3^+*x*^2^+*x*+1
*x* ^216^	195	*x* ^7^+*x*^6^+*x*+1
*x* ^217^	155	*x* ^7^+*x*^4^+*x*^3^+*x*+1
*x* ^218^	43	*x* ^5^+*x*^3^+*x*+1
*x* ^219^	86	*x* ^6^+*x*^4^+*x*^2^+*x*
*x* ^220^	172	*x* ^7^+*x*^5^+*x*^3^+*x*^2^
*x* ^221^	69	*x* ^6^+*x*^2^+1
*x* ^222^	138	*x* ^7^+*x*^3^+*x*
*x* ^223^	9	*x* ^3^+1
*x* ^224^	18	*x* ^4^+*x*
*x* ^225^	36	*x* ^5^+*x*^2^
*x* ^226^	72	*x* ^6^+*x*^3^
*x* ^227^	144	*x* ^7^+*x*^4^
*x* ^228^	61	*x* ^5^+*x*^4^+*x*^3^+*x*^2^+1
*x* ^229^	122	*x* ^6^+*x*^5^+*x*^4^+*x*^3^+*x*
*x* ^230^	244	*x* ^7^+*x*^6^+*x*^5^+*x*^4^+*x*^2^
*x* ^231^	245	*x* ^7^+*x*^6^+*x*^5^+*x*^4^+*x*^2^+1
*x* ^232^	247	*x* ^7^+*x*^6^+*x*^5^+*x*^4^+*x*^2^+*x*+1
*x* ^233^	243	*x* ^7^+*x*^6^+*x*^5^+*x*^4^+*x*+1
*x* ^234^	251	*x* ^7^+*x*^6^+*x*^5^+*x*^4^+*x*^3^+*x*+1
*x* ^235^	235	*x* ^7^+*x*^6^+*x*^5^+*x*^3^+*x*+1
*x* ^236^	203	*x* ^7^+*x*^6^+*x*^3^++*x*+1
*x* ^237^	139	*x* ^7^+*x*^3^++*x*+1
*x* ^238^	11	*x* ^3^+*x*+1
*x* ^239^	22	*x* ^4^+*x*^2^+*x*
*x* ^240^	44	*x* ^5^+*x*^3^+*x*^2^
*x* ^241^	88	*x* ^6^+*x*^4^+*x*^3^
*x* ^242^	176	*x* ^7^+*x*^5^+*x*^4^
*x* ^243^	125	*x* ^6^+*x*^5^+*x*^4^+*x*^3^+*x*^2^+1
*x* ^244^	250	*x* ^7^+*x*^6^+*x*^5^+*x*^4^+*x*^3^+*x*
*x* ^245^	233	*x* ^7^+*x*^6^+*x*^5^+*x*^3^+1
*x* ^246^	207	*x* ^7^+*x*^6^+*x*^3^+*x*^2^+*x*+1
*x* ^247^	131	*x* ^7^+*x*+1
*x* ^248^	27	*x* ^4^+*x*^3^+*x*+1
*x* ^249^	54	*x* ^5^+*x*^4^+*x*^2^+*x*+1
*x* ^250^	108	*x* ^6^+*x*^5^+*x*^3^+*x*^2^
*x* ^251^	216	*x* ^7^+*x*^6^+*x*^4^+*x*^3^
*x* ^252^	173	*x* ^7^+*x*^5^+*x*^3^+*x*^2^+1
*x* ^253^	71	*x* ^6^+*x*^2^+*x*+1
*x* ^254^	142	*x* ^7^+*x*^3^+*x*^2^+*x*
*x* ^255^	1	1

**Table 2:** S-box in the form of 16 × 16 matrix.

135	225	225	71	210	134	105	135	62	188	139	181	160	242	34	194
179	119	182	126	107	129	222	232	57	126	147	0	119	181	34	105
62	42	164	75	204	221	181	111	222	19	111	45	197	35	132	210
108	186	73	44	181	171	51	134	77	188	63	107	46	81	119	47
192	88	134	172	248	94	119	242	240	221	174	57	17	242	253	17
165	135	237	215	98	24	8	208	74	134	192	210	239	171	72	142
177	158	247	147	246	148	12	71	251	254	107	181	51	213	121	164
143	132	88	160	253	223	36	34	215	252	13	244	33	120	15	179
73	33	232	125	36	223	126	80	2	17	47	172	225	1	200	235
171	160	254	80	144	252	246	200	232	235	46	52	120	246	106	219
15	173	95	14	108	245	95	74	160	240	25	120	33	252	72	208
14	239	64	138	141	8	212	12	3	106	197	125	204	25	232	35
225	248	108	120	60	17	242	250	90	36	17	34	77	42	237	194
81	148	177	108	212	52	212	81	247	100	64	24	38	244	77	174
235	252	60	210	213	208	139	129	45	219	33	98	138	201	7	141
38	188	181	165	208	121	2	126	140	171	13	188	182	36	250	143

**Table 3:** S-box in the form of 16 × 16 matrix.

169	36	36	188	89	218	26	169	222	165	66	49	230	176	78	50
75	147	98	102	104	23	138	247	186	6	41	0	147	49	78	26
222	181	198	15	22	69	49	206	138	90	206	193	141	156	184	89
208	11	202	238	49	179	10	218	60	165	161	104	159	231	147	35
130	254	218	123	27	113	147	176	44	69	241	186	152	247	71	152
145	169	139	239	67	143	29	81	137	218	130	89	22	179	101	42
219	183	131	41	233	82	205	188	216	142	104	49	10	242	118	198
84	184	254	230	71	9	37	78	239	173	135	250	39	59	38	75
202	39	247	51	37	9	102	102	4	152	35	123	36	5	28	235
179	230	1	253	168	173	207	28	247	235	159	20	59	207	52	86
38	246	226	19	208	233	226	137	230	44	3	59	39	173	101	81
19	22	95	33	21	29	121	205	99	52	141	51	221	3	247	156
36	27	208	59	185	152	176	108	223	37	152	78	60	181	139	50
231	82	219	208	121	20	121	231	131	17	95	143	148	250	60	241
235	173	185	89	242	81	66	23	193	86	39	67	33	56	100	21
148	165	49	145	81	118	4	102	132	179	135	65	98	37	108	84

**Table 4:** S-box in the form of 16 × 16 matrix.

69	222	6	216	134	50	52	69	94	3	222	210	167	168	88	146
186	65	249	89	213	97	83	29	244	46	174	234	65	139	108	52
162	157	199	189	102	118	87	122	83	69	122	19	152	198	19	116
18	234	252	173	87	102	63	50	136	3	159	159	171	80	149	66
218	98	166	109	192	86	149	61	20	118	213	244	33	61	12	228
176	135	190	111	141	220	61	115	171	174	218	1	154	60	220	8
202	86	249	174	19	176	177	216	113	202	143	210	63	44	135	199
228	19	98	203	12	217	57	88	111	181	14	250	176	179	94	186
45	176	89	230	203	217	89	90	42	33	66	190	6	121	6	69
102	167	202	90	159	191	49	6	175	208	171	185	155	7	146	193
94	183	205	170	18	19	205	171	203	20	156	179	192	181	220	115
170	32	102	72	161	61	115	177	121	188	152	230	102	156	89	198
182	192	106	155	129	113	168	233	189	203	228	108	136	157	190	146
184	176	202	106	160	185	160	80	11	37	102	220	254	250	173	213
208	191	129	134	44	198	222	97	19	193	192	141	72	59	148	161
254	137	139	176	198	159	42	46	37	60	44	137	249	57	233	230

**Table 5:** S-box in the form of 16 × 16 matrix.

47	138	64	195	218	5	20	47	113	8	138	89	126	252	254	154
110	190	54	225	242	175	187	48	250	159	241	251	190	66	208	20
191	213	14	87	68	199	127	236	187	47	236	90	73	7	90	248
45	251	173	246	127	68	161	5	79	8	115	115	179	253	164	97
43	67	163	174	130	177	164	111	180	199	242	250	39	111	205	61
227	169	174	206	21	172	111	124	179	241	43	2	57	185	69	29
112	177	54	241	90	227	219	195	31	112	84	89	161	238	169	14
61	90	67	224	205	155	186	254	206	49	19	108	227	75	113	110
193	227	225	244	224	155	225	223	181	39	97	174	64	118	64	47
68	126	112	223	115	65	133	64	253	81	179	55	114	9	154	25
113	196	167	215	45	90	167	179	224	180	228	75	130	49	172	124
215	157	68	101	209	111	124	219	118	98	73	241	68	228	225	7
98	130	52	114	23	31	252	243	87	241	61	208	79	213	174	154
196	227	112	52	230	55	230	253	232	74	68	172	142	108	246	242
81	130	23	218	238	7	138	175	90	25	130	21	101	210	82	209
1	66	158	227	7	115	181	159	74	185	238	158	54	186	243	244

**Table 6:** S-box in the form of 16 × 16 matrix.

14	131	198	2	103	102	227	14	219	187	162	18	206	88	163	75
234	130	85	242	138	232	61	60	157	122	170	17	130	65	70	227
219	172	182	182	22	192	7	235	61	36	231	37	111	96	160	253
2	17	26	70	7	47	235	249	86	187	104	5	160	21	27	232
243	117	54	237	146	24	27	175	58	215	54	157	16	175	187	55
39	5	73	161	30	130	84	187	74	54	143	253	65	26	218	75
4	24	175	170	177	33	152	2	51	213	138	18	235	124	5	182
59	160	117	188	187	152	145	163	161	124	160	142	131	55	193	20
26	131	230	159	52	152	242	115	45	16	232	237	198	169	133	36
47	206	32	115	5	166	177	133	60	43	160	153	6	177	254	45
193	2	140	191	197	70	114	74	188	58	242	55	9	124	218	187
191	65	145	157	212	84	75	152	169	254	111	159	22	242	230	96
131	146	134	6	183	51	88	171	182	52	55	130	86	172	202	75
2	33	4	134	25	153	37	21	175	19	145	130	67	142	70	54
43	166	183	103	7	225	162	242	37	45	141	30	157	183	183	212
67	32	65	39	225	104	10	171	46	26	160	32	85	145	171	59

**Table 7:** S-box in the form of 16 × 16 matrix.

19	92	7	4	136	68	144	19	86	220	191	45	83	254	99	15
251	46	214	176	33	247	111	185	213	236	215	152	46	190	94	144
86	123	98	98	234	130	128	235	111	37	245	74	206	217	230	71
4	152	6	94	128	35	235	54	177	220	13	32	230	117	12	247
125	237	80	139	154	143	12	255	105	239	80	213	76	255	220	160
53	32	202	209	96	46	107	220	137	80	84	71	190	6	43	15
16	143	255	215	219	39	73	4	10	242	33	45	235	151	32	98
210	230	237	165	220	73	77	99	209	151	230	42	92	160	25	180
6	92	244	115	26	73	176	124	193	76	247	139	7	229	109	37
35	83	157	115	5	166	177	133	60	43	160	153	213	6	177	254
45	193	4	132	65	141	94	62	137	165	105	176	160	0	151	43
220	65	190	77	213	121	107	30	73	229	1	206	115	234	176	244
217	92	154	218	64	196	10	254	179	98	20	160	46	177	123	112
15	4	39	218	50	146	49	117	255	2	77	46	194	42	94	80
119	63	196	136	128	36	191	176	74	193	6	96	213	196	196	121
194	157	190	53	36	13	116	179	159	6	230	157	214	77	179	210

**Table 8:** S-box in the form of 16 × 16 matrix.

94	143	242	59	55	207	84	180	238	15	216	174	179	241	214	9
44	100	118	62	11	190	13	185	63	74	132	81	193	95	57	49
244	189	158	194	237	141	69	121	232	12	199	172	90	51	203	20
128	245	58	252	119	85	101	221	48	30	51	254	111	112	188	100
162	150	37	145	27	19	67	50	94	123	168	215	28	12	167	9
45	4	240	196	35	182	244	214	70	223	169	210	213	196	62	121
211	196	82	72	158	215	202	229	48	189	217	63	62	48	137	192
53	196	98	65	161	223	85	34	194	222	58	176	59	170	94	203
30	83	63	152	3	103	175	110	99	87	205	87	29	25	162	94
105	208	148	109	86	147	43	246	34	5	49	184	251	69	24	249
121	243	151	63	241	114	196	252	66	204	0	58	136	12	180	217
16	99	106	175	196	211	210	79	92	187	229	162	33	107	207	87
126	251	237	197	216	131	220	239	183	205	183	248	29	96	217	209
230	31	126	46	252	112	215	14	162	196	212	190	120	22	243	128
113	115	89	131	114	50	241	186	53	42	161	41	14	2	2	220
31	83	1	98	108	172	169	71	20	88	87	48	101	47	99	10

**Table 9:** S-box in the form of 16 × 16 matrix.

113	84	176	210	160	166	107	150	11	38	195	241	75	88	249	58
238	17	199	222	99	174	135	55	161	137	184	231	25	226	186	140
250	87	183	50	139	21	47	118	247	205	14	123	223	10	224	180
33	233	105	173	147	214	34	69	70	96	10	1	206	129	165	17
191	85	74	77	12	90	194	5	113	197	252	239	24	205	126	58
193	16	44	200	156	98	250	249	94	9	229	89	242	200	222	118
178	200	211	101	183	239	112	122	70	87	155	161	222	70	158	130
40	200	67	190	209	9	214	78	50	138	105	227	210	215	113	224
96	187	161	73	8	136	255	103	134	127	167	127	48	3	191	113
26	81	82	189	177	41	119	207	78	32	140	149	216	47	143	54
118	125	170	161	88	62	200	173	97	221	1	105	79	205	150	155
76	134	52	255	200	178	89	240	91	220	122	191	39	104	166	127
102	216	139	141	195	92	172	22	196	167	196	27	48	217	155	162
244	192	102	159	173	129	239	19	191	200	121	174	59	234	125	133
31	124	225	92	62	5	88	110	40	181	209	212	19	4	4	172
192	187	2	67	208	123	229	188	180	254	127	70	34	35	134	80

**Table 10:** S-box in the form of 16 × 16 matrix.

30	245	179	8	179	0	131	143	253	100	175	140	18	95	38	245
213	252	192	120	233	138	148	89	55	11	249	230	180	123	187	172
91	127	197	228	26	243	180	81	116	210	36	195	186	20	232	104
161	30	186	135	163	173	160	48	247	75	240	7	186	181	38	201
186	249	152	220	223	7	94	170	217	30	39	92	206	162	160	163
43	0	103	195	163	204	184	119	159	3	207	75	109	131	27	207
135	231	246	80	10	127	27	97	211	73	97	238	76	188	70	77
17	47	179	249	187	177	227	44	197	71	29	72	159	234	136	34
118	63	109	61	68	70	175	217	41	75	34	238	214	74	94	157
166	155	29	171	34	1	20	14	190	91	196	26	8	162	181	132
33	159	2	131	151	160	153	118	195	89	140	200	23	25	63	174
82	63	190	210	23	218	148	171	12	42	158	203	15	85	32	28
176	156	12	2	235	213	1	62	169	219	172	125	76	130	4	158
137	200	126	227	41	52	96	111	32	36	243	38	187	3	62	31
44	186	223	107	218	112	141	71	176	251	5	194	84	171	134	151
215	132	186	12	254	155	9	186	14	131	105	100	144	236	145	19

**Table 11:** S-box in the form of 16 × 16 matrix.

96	233	75	29	179	1	92	84	71	17	255	132	45	226	148	233
249	173	130	59	243	33	82	225	160	29	108	244	150	197	220	123
163	204	141	61	6	125	150	231	248	89	37	100	110	180	247	13
63	96	110	169	99	246	230	70	131	15	88	128	110	49	148	56
110	54	73	172	9	128	113	215	155	96	53	91	83	191	230	99
119	1	136	100	99	221	149	147	115	8	166	15	189	92	12	166
169	245	207	253	116	204	12	175	178	202	175	11	30	165	94	60
152	35	75	54	220	219	144	238	141	188	48	101	115	251	79	78
199	161	189	111	153	94	255	155	212	15	78	11	249	137	113	213
63	114	48	179	78	2	180	19	174	163	200	6	29	191	49	184
39	115	4	92	170	230	146	199	100	225	132	28	201	3	161	241
211	161	174	89	201	43	82	179	205	181	183	224	38	214	157	24
227	228	205	4	235	242	161	229	86	123	51	30	46	16	183	158
28	102	144	212	5	217	206	157	37	125	148	220	8	222	192	238
110	9	104	43	129	31	21	188	227	216	32	50	107	179	218	170
239	184	110	49	142	114	50	110	19	92	26	17	168	203	77	23

**Table 12:** Assessment of nonlinearity.

S-boxes	Nonlinearity
Transformed S-box	107.3
APA S-box [25]	112
*S*_8_ Liu J S-box [26]	104.87
Hussain et al. [27]	104.75
Residue prime [28]	99.5

**Table 13:** Comparison of strict avalanche criterion.

S-boxes	Max. value	Min. value
Transformed S-boxes	0.61	0.57
APA S-box [25]	0.56	0.437
S_8_ Liu J S-box [26]	0.59	0.429
Hussain et al. [27]	0.59	0.391
Residue prime [28]	0.67	0.343

**Table 14:** Assessment of BIC.

S-boxes	Min. value
Transformed S-box	101.3
APA S-box [25]	112
*S*_8_ Liu J S-box [26]	99
Hussain et al. [27]	100
Residue prime [28]	94

**Table 15:** Analysis of LP.

S-boxes	Max. value
Transformed S-box	0.15
APA S-box [25]	0.062
*S*_8_ Liu J S-box [26]	0.105
Hussain et al. [27]	0.125
Residue prime [28]	0.132

**Table 16:** Analysis of DP.

S-boxes	Max. DP
Transformed S-box	0.06
APA S-box [25]	0.0156
*S*_8_ Liu J S-box [26]	0.0390
Hussain et al. [27]	0.125
Residue prime [28]	0.281

**Table 17:** Comparison of MLC.

S-boxes	Entropy	Contrast	Correlation	Energy	Homogeneity
Host image [23]	7.6062	0.4896	0.9075	0.0785	0.8009
Proposed S-box	7.9972	11.2629	−0.0039	0.0159	0.3855
AES	7.73018	7.322085	0.087904	0.024477	0.483523
APA [29]	7.688383	7.736859	0.216816	0.022942	0.486265
Prime [26]	7.65955	6.368367	0.099634	0.026099	0.49848
Skipjack [31]	7.673853	6.805101	0.195849	0.026131	0.495087

## Data Availability

No data were used to support the findings of this study.
